# Optimizing Residual Networks and VGG for Classification of EEG Signals: Identifying Ideal Channels for Emotion Recognition

**DOI:** 10.1155/2021/5599615

**Published:** 2021-03-30

**Authors:** Kit Hwa Cheah, Humaira Nisar, Vooi Voon Yap, Chen-Yi Lee, G. R. Sinha

**Affiliations:** ^1^Department of Electronic Engineering, Faculty of Engineering and Green Technology, Universiti Tunku Abdul Rahman, Kampar 31900, Malaysia; ^2^Department of Electronics Engineering and Institute of Electronics, National Chiao Tung University, Hsinchu, Taiwan; ^3^Myanmar Institute of Information Technology (MIIT), Mandalay, Myanmar

## Abstract

Emotion is a crucial aspect of human health, and emotion recognition systems serve important roles in the development of neurofeedback applications. Most of the emotion recognition methods proposed in previous research take predefined EEG features as input to the classification algorithms. This paper investigates the less studied method of using plain EEG signals as the classifier input, with the residual networks (*ResNet*) as the classifier of interest. *ResNet* having excelled in the automated hierarchical feature extraction in raw data domains with vast number of samples (e.g., image processing) is potentially promising in the future as the amount of publicly available EEG databases has been increasing. Architecture of the original *ResNet* designed for image processing is restructured for optimal performance on EEG signals. The arrangement of convolutional kernel dimension is demonstrated to largely affect the model's performance on EEG signal processing. The study is conducted on the Shanghai Jiao Tong University Emotion EEG Dataset (SEED), with our proposed *ResNet18* architecture achieving 93.42% accuracy on the 3-class emotion classification, compared to the original *ResNet18* at 87.06% accuracy. Our proposed *ResNet18* architecture has also achieved a model parameter reduction of 52.22% from the original *ResNet18*. We have also compared the importance of different subsets of EEG channels from a total of 62 channels for emotion recognition. The channels placed near the anterior pole of the temporal lobes appeared to be most emotionally relevant. This agrees with the location of emotion-processing brain structures like the insular cortex and amygdala.

## 1. Introduction

Emotion is the conscious or subconscious neuropsychological response generated upon external or internal stimuli which are of major concern to the person.

Emotion involves the interrelated synchronization of a number of organismic subsystems encompassing the central nervous system, the autonomous nervous system, the neuroendocrine system, the somatic nervous system, and the conscious or subconscious reactions of the respective effectors [1].

Expression of emotion includes the linguistic choice of words, speaking rate, intonation, facial expression, gesture, and posture. Emotion can also be reflected via the autonomous nervous system and neuroendocrine system into the cardiovascular dynamics [2, 3], respiratory patterns [4], and electrodermal activity [5]. Nevertheless, all the peripheral emotion reactions arise from the neurological activities in the brain. The cerebral neuronal activities can be recorded as the electrical potentials on the scalp with the electroencephalography (EEG) technique [6].

Emotion recognition algorithms are useful in human-machine interaction, allowing machines to identify the emotional or affective mental states of humans [7]. Affective computing [8] and the “empathetic” capability of the machine can have an important role in the development of many applications such as neurofeedback therapies for mood and cognition improvement [9]. Also, affective computing has substantial potential in helping victims with a neurodevelopmental disorder and improving their ability to emote and identify emotional expressions [10].

Emotion recognition can be achieved by analyzing the abovementioned nonphysiological expression such as the vocal signals, facial expression and bodily gestures, and the physiological signals such as the photoplethysmogram (PPG), electrocardiogram (ECG), electrodermal activity (EDA), electromyogram (EMG), and electroencephalogram (EEG).

Emotion recognition methods can be classified as multimodal or single modal. The combined information from two or more of the physiological and nonphysiological aspects is required in the multimodal emotion recognition methods, while the single-modal recognition approach typically utilizes one type of physiological signal. EEG is among the most widely used single-modal signal for emotion recognition as it carries the information of the brain neuronal activities from which almost all other physiological and nonphysiological reactions arise [11–14].

A recent extensive 5-year review by Craik et al. (2019) [15] on the current research state of deep neural networks for EEG classification reported the finding of only about 22% of the emotion recognition research using EEG signal values as the input data, with the remaining vast majority using the precalculated EEG features or images constructed from the EEG features as the input data to the classifiers.

Another 8-year review (2010–2018) by Roy et al. (2019) [16] on deep learning architectures for EEG analysis covering 154 publications reported that only about 12% of the deep learning architectures used for the affective mental domain were the convolutional neural networks (CNNs).

In recent years, there are an increasing number of publicly shared EEG databases among the research community. With this trend ongoing, increasingly sufficient variations of input EEG samples will be available soon for the training of very-deep neural networks. The projected future availability of sufficiently large variation of input EEG samples can promisingly solve the problem of overfitting of very-deep neural networks to the small research pool of EEG samples which are currently insufficient to serve as a good representative of the population. Therefore, our work studies the application of variants of very-deep CNN (*ResNet18* and *VGG16*) on the plain EEG signal (instead of precalculated EEG features) classification, with emotion recognition as the case study. We will present the architectural optimization of Residual Network (*ResNet*) for EEG signal classification. The performance of the variants of *ResNet* will be compared with the *VGG* variants. We will also compare the significance of different EEG channel subsets for emotion recognition and present the relevance of different subsets of EEG channels to emotion recognition.

## 2. Methodology

### 2.1. Experiment Design of SEED Dataset

This study uses the EEG signals recorded in the SEED experiment by the Shanghai Jiao Tong University (SJTU). The SEED dataset [17, 18] is an emotion-related EEG dataset publicly available for research purposes. The stimuli in the SEED experiment were 15 film clips carefully chosen such that each elicits a single desired target emotion. Each film clip lasts about 4 minutes and is coherent to either positive, neutral, or negative valence emotion as described in Table 1.

SEED experiment had 15 participants. Every participant underwent 3 sessions of the experiment, with at least one-week interval between every 2 sessions. Each experiment session contained 15 trials, each playing one of the 15 film clips followed by self-assessment and a short rest.  Figure 1 shows the structure of the experiment session.

The play sequence of the film clips was arranged such that no two consecutive trials carried the clips of the same emotion category.

The EEG signals were recorded with 62 active AgCl electrodes of the ESI NeuroScan System at a sampling frequency of 1000 Hz. The electrode placement was based on the international 10–20 system as shown in Figure 2.

The recorded EEG signals were then downsampled to 200 Hz and a bandpass frequency filter of 0.5 Hz to 70 Hz was applied.

### 2.2. SEED Dataset Literature Review

The research working on the SEED dataset in the recent three years (2018–2020) was reviewed and is summarized in Table 2. Although many of the research works were using one or another kind of neural network classifier, almost all of the attention had been placed on using manually extracted EEG features, instead of plain EEG signals.

Using plain EEG signals as the input data to the emotion classifiers has currently received relatively much lower research attention. Although the number of currently available public EEG research databases may not yet be sufficiently representative of the general population, the trend of an increasing number of publicly available EEG databases shall warrant more research works into the application of very-deep neural networks on plain EEG signals.

In line with this, the focus of this work is on eliciting the architectural modification on the original image-oriented *ResNet* and *VGG* that results in a vast improvement of their performance on plain EEG signal. In addition, we have also proposed the location of EEG channels that are most useful for emotion recognition.

### 2.3. EEG Dataset Preprocessing

As the target emotion caused by watching the film clip would not likely be successfully induced immediately at the start of the film clip, we have set a buffering period of 90 seconds for the emotion establishment. Therefore, the initial 90 seconds of each of the 4-minute EEG trials were discarded.

The remaining EEG recording is split into 2-second nonoverlapping segments, with each EEG segment assuming the length of 400 sampling points for the sampling frequency of 200Hz. Each of the nonoverlapping segments is then normalized along the time axis, respectively, using the Euclidean normalization method. All the generated EEG segments are split into five subpools for 5-fold cross-validation of the model performance.

### 2.4. Optimizing *ResNet* and *VGG* for EEG Signals

Figures 3 and 4, respectively, illustrate the architectural details of different versions of *ResNet18* and *VGG16* examined in this study.

#### 2.4.1. *ResNet* Optimization

The original architecture of *ResNet18* consisting of 17 convolutional layers and 1 layer of the fully connected network is depicted in Figure 3(a).

As the original *ResNet18* is designed for image processing, the convolutional kernels within the model are all 2-dimensional kernels. It has 3-by-3 kernels throughout its convolutional path, except for the very first convolutional layer (*Conv 0*) which has 7-by-7 kernels.

The color coding of Figure 3 denotes the major convolutional blocks of the ResNet. The convolutional layers of the same color have the same number of kernels (e.g., orange for 64 kernels, yellow for 128 kernels, green for 256 kernels, and blue for 512 kernels). The darker color layers are convolutional layers, while the lighter layers are the other functional layers in the block, such as the batch normalization (BN) function, the Rectified Linear Unit (ReLU) activation function, the summation (Sum) of the by-passed feature map and the main convolution feature map, and the adaptive average pooling (AvgPool). The adaptive AvgPool layer before the fully connected (FC) layer allows the model to process EEG signals of different numbers of channels without the need to reassign the number of connections in the FC network.

The last layer of the *ResNet18* is a single layer of a fully connected (FC) network with three output nodes, corresponding to the three emotion classes.

There are two types of bypass connection in the ResNet, i.e., the identity bypass and the downsampling bypass. The identity bypass has its feature map being passed on, skipping two convolutional layers without any further processing before the summation function. The downsampling bypass happens at the initial stage of every major convolutional block, where the input feature maps will have their map size reduced due to kernel stride and the number of feature maps will increase due to the increment of convolutional kernels. Therefore, the downsampling bypass is necessary in order to have the dimension of the shortcut data matching the data dimension of the main convolutional path. While the identity bypass performs no additional processing on the data passed onwards, the downsampling bypass has 1-by-1 convolutional kernels which introduce an additional small number of trainable parameters as reported in Figure 3.

In this study, three variants of the original *ResNet18* were constructed and investigated. Two of the three *ResNet18* variants are illustrated in Figures 3(b) and 3(c). The 2D kernels of the *ResNet* were all restructured into 1D kernels along either the temporal(time)-dimension or the spatial(channel)-dimension.

The variant in Figure 3(b) has alternating temporal and spatial-dimension convolution. Eckart and Young [28] and Maji and Mullins [29] reported that the matrix such as the convolution filters can be well approximated with an arbitrary number of lower rank matrices. Maji and Mullins (2018) [29] had also demonstrated the feasibility of separating the 2D kernels of the well-established CNNs (e.g., *AlexNet*, *VGG-16*, *Inception-v1*, *ResNet-152*) into alternating 1D vertical and horizontal kernels, achieving near baseline accuracy for image classification with a significant speedup of training.

Nevertheless, given the different format and nature of EEG signals from the images, the alternating arrangement of 1D horizontal (time-dimension) kernel and 1D vertical (spatial-dimension) kernel may not be the optimal design for EEG signal processing. Therefore, we have constructed another variant of *ResNet18* (Figure 3(c)) with the initial two major convolutional blocks (all the nine initial convolutional layers) operating purely in the temporal dimension before introducing the spatial convolutional kernels. The spatial-dimension convolution of this *ResNet* variant appears only in the final two convolutional blocks.

In addition, we have investigated the effect of initializing the convolutional path with spatial-dimension convolution, by making only a single change in the initial layer (*Conv 0*) of *ResNet18-1D-kernel-(T-S-alternate)* in Figure 3(b), from time-dimension convolution into spatial-dimension convolution. We have name-coded this variant as *ResNet18-1D-kernel-(S-T-alternate)*, for comparison with the model in Figure 3(b) to highlight the great impact of the abovementioned single minor architectural change on the model's performance which is presented in Figure 5.

The right columns of the Figures 3(a)–3(c) indicate the number of trainable parameters in each architectural layer of the *ResNet* variants.

#### 2.4.2. *VGG* Optimization

As illustrated in Figure 4, variants of *VGG16* are also constructed for performance comparison with the variant of *ResNet18*. The *VGG* models have classical convolutional pathways without data bypassing. The *VGG16* has five major convolutional blocks, with two convolutional layers in each of its first two major convolutional blocks and three convolutional layers in each of its last three convolutional blocks. These thirteen convolutional layers together with the final three FC layers have made up the 16 main functional layers in the *VGG16*.

Figure 4(a) shows the structure of the *VGG16* with all the original 2D kernels being modified into 1D kernels along either the temporal or spatial dimension. The model in Figure 4(b) is named *VGG14-1D* with the removal of the two hidden FC layers from the *VGG16-1D*, such that the fully connected network is more closely resemble and comparable to that of the *ResNet18*.

The *VGG* architectures in Figure 4 are color-coded such that the transition between different color blocks is preceded by max-pooling (*MaxPool*) operation along the dimension of the previous convolution operation. The adaptive *AvgPool* layer before the FC networks is for the same purpose as described for the *ResNet18*.

We have also investigated the importance of batch normalization in CNN for EEG processing by removing the BN layers of the *VGG16* as in Figure 4(c). The performance analysis is presented in the Results section.

### 2.5. Model Training

The objective function for model optimization during training was set as the cross-entropy loss of the CNN outputs. Adam optimizer was used to update the trainable parameters of the CNN at the learning rate of 0.001, based on the backpropagated error from the output cross-entropy loss.

The model training process was conducted with stochastic minibatches, with the size of each minibatch being one 200^th^ of the total training pool. Thus, one complete training epoch consists of 200 training iterations. The training data pool will be reshuffled after every complete training epoch to ensure the different combinations of minibatch samples in the subsequent training epochs. Stochastic minibatch training serves to prevent the training process from being stuck at the local minima of the objective function.

## 3. Results and Discussion

### 3.1. Variants of *ResNet18*

Figure 5 presents the averaged 5-fold cross-validation classification accuracy of the ResNet variants, using different subsets of EEG channels as their data input.

The *ResNet* variant with 1D kernels has generally outperformed the original ResNet18, particularly in the scenario of using a lower number of EEG channels (10 channels for each subset). Not only has the classification improved with the *ResNet18* architectural restructuring from 2D-kernel convolution to 1D-kernel convolution, the total number of trainable parameters (obtainable by summing up the layer-wise parameters in Figure 3) in the *ResNet18* has also seen a reduction of more than 50% from the original 11.17 million parameters down to the range of 4.27 to 5.34 million parameters.

As pointed out in Section IV-B, the models *ResNet18-1D-(S-T-alternate)* and *ResNet18-1D-(T-S-alternate)* differ in only their very first convolutional layer (the *Conv-0* of Figure 3(b)), where the *ResNet18-1D-(T-S-alternate)* model has *Conv-0* as temporal convolution while the *ResNet18-1D-(S-T-alternate)* model has its *Conv 0* as spatial convolution. Although this single change in *Conv-0* has resulted in the difference in parameter count by only 256 ((1 × 9 ‒ 5 × 1) × 64 = 256), the performance in EEG signal classification has seen substantial improvement by about 10% elevation (using either all 62 channels, the outermost 10 channels, or outer 10 channels), as presented in Figure 5. This strongly indicates that the convolution operation on plain EEG signal should not be initiated with spatial(channel)-dimension convolution.

Some other previous works that used CNN for plain EEG signal processing had also forced the convolution process to operate only along either the temporal or spatial dimension for every single convolutional layer. Most of the works [30–36] applying 1D-kernel CNN on EEG signals had initiated the convolutional path with temporal convolution. However, they had not provided the performance comparison with the models that did otherwise, as we highlighted in this study.

We took a further step of increasing the number of layers of pure temporal convolution before starting spatial convolutional operation, as in the architecture of *ResNet18-1D-(T-then-S)* in Figure 3(c). The *ResNet18-1D-(T-then-S)* model has outperformed all the other *ResNet18* variants substantially, in every classification scenario as reported in Figure 5.

This supports that constructing multiple consecutive layers of temporal convolution before starting spatial convolution is beneficial for extracting distinctive information from the EEG signals. Although *ResNet* had been reported with inferior performance than the typical CNN at EEG classification in [34], their *ResNet* architecture was, however, designed with spatial convolution very early on as the second convolutional layer. If more temporal convolutional layers were introduced before the spatial convolution, the *ResNet* presented in [34] could potentially have seen significant performance improvement.

With the presence of multiple consecutive temporal convolutional layers before spatial convolution, higher hierarchical features within each EEG channel could be extracted before comparing across different channels. Direct cross-channel convolution of rudimentary EEG voltages may not carry as much distinctive information as that of the higher hierarchical features.

Plain EEG signals carry only voltage levels measured over the scalp. Every single sampling point of the voltage level in an EEG channel is not as meaningful as a sequence of sampling points along the channel. The excessively short receptive field over a single channel is susceptible to recording artifacts and other nonessential signal variations.

Therefore, with multiple consecutive temporal convolutional layers, the initial stages of the model can cover a larger receptive field over the raw signal, at the same time extracting features of a higher level of abstraction from the particular channel. Comparing the rudimentary EEG signal sampling point by sampling point across the channels may have considerably taken into account the undesired meaningless voltage variations, resulting in lower classification accuracy in the *ResNet18-1D-(S-T-alternate)* model.

We have also constructed and examined another variant of the *ResNet18-1D-(S-then-T)* model with its several initial convolutional layers all being spatial-dimension convolution followed by temporal convolution only. This model which was not presented in Figure 3 had presented worse performance than even the *ResNet18-1D-(S-T-alternate)* model, which further supports the proposal above that EGG signal convolution for emotion recognition should ideally be started with temporal-dimension convolution.

Figure 6 reports the training-validation performance log of the four variants of *ResNet-1D*, using the 10 outermost channels. Based on the training-validation cross-entropy loss plot, the *ResNet18-1D-(T-then-S)* model, which had outperformed all the rest, was clearly less susceptible to overfitting. The other three *ResNet18-1D* models all had started to experience overfitting after around eight to ten training epochs, with the models *ResNet18-1D-(S-then-T)* and *ResNet18-1D-(S-T-alternate)* experiencing the greatest degree of overfitting.

### 3.2. *ResNet* versus *VGG*

We have compared the performance of *ResNet18* with the more classical CNN architecture (the *VGG16*) from the aspects of classification accuracy, the number of trainable parameters, and the model training convergence speed.

Figure 7 shows that the classification accuracy achieved by *ResNet18-1D(T-then-S)*, *VGG14-1D*, and *VGG16-1D* models is very close to each other. The *ResNet18-1D(T-then-S)* achieves 93.42% classification accuracy, outperforming the *VGG* at using all 62 EEG channels. The *VGG* models have achieved higher accuracy at the less significant subsets of EEG channels (e.g., using the innermost 10 channels).

Given the almost negligible difference in the classification accuracy, the *ResNet18-1D(T-then-S)* model contains only 5.34 million parameters, which is only about 36.3% of that in the *VGG14-1D* model which has 14.72 million parameters. The *VGG16-1D* has an even staggering greater number of parameters (at 46.18 million) due to a large number of fully connected perceptrons in its original 3-layer FC networks. This densely connected FC network containing over 31 million parameters does not appear to be essential to the classification accuracy.

Another aspect of performance measurement investigated is the convergence speed of the model under training. With reference to Table 3, using all 62 EEG channels, the *ResNet18-1D(T-then-S)* and the *VGG14-1D* models are able to converge to above 95% training accuracy in 11 epochs and 10 epochs, respectively. The *VGG16-1D* requires a greater number of training epochs (14 complete rounds) to reach its training accuracy of 95%. The lower convergence speed of *VGG16-1D* is likely due to its complex FC network.

The *ResNet18-1D(T-then-S)* model completes a training epoch with (1665/11 ≈ 151) seconds, while the *VGG* models require a much greater amount of time to complete a training epoch (*VGG14-1D* using about 249 seconds, and *VGG16-1D* using about 250 seconds).

Similarly, the *ResNet18-1D(T-then-S)* uses only about 38 seconds for a complete training epoch with 10 EEG channels, while the two *VGG* models use about 50 seconds for completing a training epoch.

The *VGG14-1D-(no batch norm)* illustrated in Figure 4(c) is the version of *VGG14-1D* without the batch normalization function after every convolutional layer. This model without the batch normalization had failed to progress well even in its training phase. The training accuracy of this model had stayed at around 35%, with the training loss staying at around the initial value.

The failure of this *VGG14-1D-(no batch norm)* has indicated the importance of batch normalization in training deep CNN on EEG signals, even with the EEG signals being prenormalized before being passed into the CNN model. All the *ResNet18* variants in Figure 3 are also equipped with batch normalization at the output of their convolutional layers.

In our model, each layer of the batch normalization function introduces two additional trainable parameters per feature map. The dimension of the feature map depends on the number of convolutional kernels immediately preceding the batch norm function.

The short EEG segments being passed into the classifier may contain large signal amplitude variations from segment to segment. Different batches of the EEG segments may also encounter the problem of large internal covariate shift [37] which is a notorious reason for the diverging loss during model optimization [38].

This does not only slow down the training speed by demanding a very low learning rate but also potentially disrupt altogether the convergence of the model optimization process as experienced in our model (Figure 4(c)) without batch normalization.

### 3.3. Channel Significance in Emotion Recognition

Identifying the most critical subsets of EEG channels can reduce the input data redundancy and ease the design and mounting of portable consumer-friendly EEG recording hardware. Therefore, previous works [39–41] had tried to identify the subsets of EEG channels that are most crucial for emotion recognition. In line with the purpose, we have looked into the emotion EEG channel significance with regard to lateral-medial placement, along the nasion-inion axis, and in terms of the left-versus-right hemispheric discrepancy.

#### 3.3.1. Electrode Distance to the Midline

With reference to Figures 5(a) and 5(b), the relevance of different subsets of EEG channels for emotion recognition is investigated, with respect to the channels' distance from the midline.

The trend of classification accuracy as reported in Figure 5 follows that the more laterally placed the EEG channels are, the higher the classification accuracy they deliver. This implies that more emotionally distinctive information is carried in the laterally placed (farther away from the midline) EEG channels than the medially placed channels.

The possible reason for this channel significance distribution pattern is that the lateral channels are in fact placed over or close to the temporal region above the ears on the scalp. These electrode locations are closer to the brain structures that are highly involved in emotional response. These structures (such as the anterior temporal pole, the insular cortex, the amygdala, and the hippocampus [42–44]) are either part of the temporal lobe itself or lying at just the medial side of the temporal lobe. Hence, the more medially placed EEG electrodes are located higher up on top of the scalp and are hence farther away from these emotionally important brain structures.

#### 3.3.2. Along the Nasion-Inion Axis

Figure 8 shows the 5-fold cross-validated emotion classification accuracy of *ResNet18-1D(T-then-S)* model, using four different subsets of EEG channels along the nasion-inion axis.

As indicated by Figure 8(b), these subsets of EEG channels, respectively, cover the frontal region (blue), centrotemporal region (green), centroparietal region (yellow), and the parietooccipital region (red).

In coherence with the distribution of emotionally important brain structures (e.g., the anterior temporal pole, the insular cortex, and the amygdala) discussed above, the three different emotion classes are best classified with the twelve centrotemporal channels (green color coded) because these twelve channels are located nearest to these structures, relative to the other three subsets.

The twelve-frontal-channel subset gives the same accuracy as the twelve parietal channels. The occipital channels are the least emotionally correlated set of EEG channels.

#### 3.3.3. Cerebral Lateralization of Emotion

Figure 9 shows the 5-fold cross-validation accuracy using EEG channels of the left hemisphere versus the right hemisphere. The left channels present around 4-5% higher accuracy than the right channels. Using only 10 lateral channels of the left hemisphere has resulted in 88.48% average accuracy which is still even better than using all 27 right-hemispheric channels which give 86.96%.

This lateralized significance of EEG channels in emotion recognition can be due to the fundamental cerebral lateralization [45, 46] or simply because of the nature of the SEED experiment design.

The stimuli of the SEED experiment were movie clips, and the mode of content delivery of movies can be heavily verbal or language-based. The center of language processing and understanding is located exactly in the lateral side of the left temporal lobe, known as Wernicke's area [47]. Therefore, the imbalanced activation of Wernicke's area in comparison to its right-hemispheric counterpart area can be a compounding factor resulting in the classification accuracy discrepancy.

#### 3.3.4. Comparing across all the Channel Subsets

Reviewing the classification results using various EEG channel subsets presented in Figures 5, 8, and 9, the ten lateral-most left and right EEG channels in Figure 5 achieved the highest accuracy (91.5%), compared to using the ten lateral left channels in Figure 9 which has achieved 88.48% recognition accuracy and the twelve centrotemporal channels in Figure 8 which have achieved 83.84% accuracy.

With a comparable number of channels used in the subsets, the above result implies that there is additional distinctive information for emotion recognition retrievable from the left-versus-right channel feature cross-correlation, in view of the pairing of 10 left and right channels giving better classification result than the 10 lateral-most left channels.

The highly emotion-correlated subsets of EEG channels identified by this work are close to the 12-channel (FT7, FT8, T7, T8, C5, C6, TP7, TP8, CP5, CP6, P7, and P8) subsets used by Zheng and Lu (2015) [41] which was reported to have achieved even higher emotion recognition accuracy than using all 62 channels.

## 4. Conclusion

This study has investigated the applicability of a very-deep convolutional neural network for plain emotion-related EEG signal classification, which is an area of relatively low research attention as most of the emotion EEG classification tasks were based on preextracted EEG features. With the future availability of a greater pool of EEG data that better represents the population, the very-deep CNNs can potentially outperform the feature-based algorithms, although they do not yet show accuracy superiority over feature-based algorithms with the current size of publicly available EEG database.

*ResNet18* and *VGG16* originally constructed for image processing were modified for EEG signal processing. The original *ResNet18* and *VGG16* designed for image processing are not ideal for direct application onto EEG signals. Our modified variants of *ResNet18* with 1D kernels have shown significant performance improvement in both the aspects of classification accuracy and reduced model parameters. The modified *ResNet18* variants have shown better training convergence speed than the *VGG16* variants.

The sequence of convolutional dimension arrangement within the *ResNet18-1D* has also been investigated for optimal EEG signal processing performance. The result findings have suggested against initiating the convolutional operation with spatial-dimension convolution. Multiple layers of consecutive temporal-dimension convolution should ideally be placed before the operation of spatial-dimension convolution. Using the SEED dataset, our best performing model [*ResNet18-1D-(T-then-S)*] has achieved a 3-class emotion classification accuracy of 93.42%.

Not of less importance, the batch normalization function proves to be essential in tackling the problem of internal covariate shift which can result in model optimization convergence failure.

Investigating the EEG channel significance for emotion recognition from the neurological aspects, the laterally placed channels around the temporal lobe show greater importance than the channels placed over other brain regions. This finding is consistent with the fact that many emotionally important brain structures are located within or nearby the temporal lobe.

## Figures and Tables

**Figure 1:** Data collection session design of SEED experiment.

**Figure 2:** EEG channel layout of SEED dataset.

**Figure 3:** Architectural details of (a) original *ResNet18* and its modified variants (b) *ResNet18-1D-kernel-*(*T-S-alternate*) and (c) *ResNet18-1D-kernel-(T-then-S*) for EEG signal processing.

**Figure 4:** Architectural details of (a) *VGG16-1D-kernel* and its modified variants (b) *VGG14-1D-kernel* and (c) *VGG14-1D-kernel (no batch norm)* for EEG signal processing.

**Figure 5:** SEED 3-class emotion recognition accuracy by variants of *ResNet18* using different subsets of EEG channels. (a) Classification accuracy and the total number of model parameters. (b) Different subsets EEG channels.

**Figure 6:** Training-validation performance log of variants of ResNet18-1D.

**Figure 7:** Classification accuracy of ResNet18-1D and VGG16 variants.

**Figure 8:** SEED 3-class emotion recognition accuracy using different subsets of EEG channels along the nasion-inion axis. (a) 5-fold cross-validation classification accuracy. (b) Electrode placement.

**Figure 9:** SEED 3-class emotion recognition accuracy comparison using left and right hemispheric EEG channels. (a) 5-fold cross-validation classification accuracy. (b) Electrode placement.

**Table 1:** Film clips in SEED dataset.

Source film name	Emotion	Number of clips
Tangshan earthquake	Negative	2
Back to 1942	Negative	3
Lost in Thailand	Positive	2
Flirting scholar	Positive	1
Just another Pandora's box	Positive	2
World heritage in China	Neutral	5

**Table 2:** Recent research on SEED dataset.

Classifier algorithm/year	Data input	Accuracy (%)
Dynamic graph CNN [19]/2018	Differential entropy (DE)	79.95
Logistic regression classifier [20]/2018	DE	72.47
GRSLR (graph regularized sparse linear regression) [21]/2018	DE, Hjorth features	88.41
Bidirectional LSTM [22]/2019	DE/Power spectral density (PSD)	94.96/86.27
Graph convolutional broad network (GCBN) [23]/2019	DE	94.24
CNN + LSTM [24]/2019	DE	89.88
Variational pathway reasoning (VPR) [25]/2019	DE	94.3
Sequential backward selection SVM [26]/2019	Hjorth features, standard deviation, sampling entropy, wavelet entropy	89
Spiking NN [27]/2020	DWT, FFT, variance	96.67

**Table 3:** Model training convergence efficiency comparison between *ResNet* and *VGG*.

	Training length to reach 95% training accuracy (epochs//seconds)	
	Using all 62 channels	Using outermost 10 channels
ResNet18-1D (T-then-s)	11//1665	11//416
VGG14-1D (T-then-s)	10//2488	10//503
VGG16-1D (T-then-s)	14//3505	12//622

## Data Availability

The data are available at http://bcmi.sjtu.edu.cn/home/seed/seed.html.

## References

[1] Scherer K. R. (2016). What are emotions? And how can they be measured?. *Social Science Information*.

[2] Sinha R., Lovallo W. R., Parsons O. A. (1992). Cardiovascular differentiation of emotions. *Psychosomatic Medicine*.

[3] Valenza G., Citi L., Lanata A., Scilingo E. P., Barbieri R. (2014). Revealing real-time emotional responses: a personalized assessment based on heartbeat dynamics. *Scientific Reports*.

[4] Homma I., Masaoka Y. (2008). Breathing rhythms and emotions. *Experimental Physiology*.

[5] Ganapathy N., Swaminathan R. (2019). Emotion recognition using electrodermal activity signals and multiscale deep convolution neural network. *Studies in Health Technology and Informatics*.

[6] Olejniczak P. (2006). Neurophysiologic basis of EEG. *Journal of Clinical Neurophysiology*.

[7] Cowie R., Douglas-Cowie E., Tsapatsoulis N. (2001). Emotion recognition in human-computer interaction. *IEEE Signal Processing Magazine*.

[8] Picard R. W. (2000). *Affective Computing*.

[9] Alkoby O., Abu-Rmileh A., Shriki O., Todder D. (2018). Can we predict who will respond to neurofeedback? A review of the inefficacy problem and existing predictors for successful EEG neurofeedback learning. *Neuroscience*.

[10] Kalantarian H., Jedoui K., Washington P. (2019). Labeling images with facial emotion and the potential for pediatric healthcare. *Artificial Intelligence in Medicine*.

[11] Hondrou C., Caridakis G. (2012). Affective, natural interaction Using EEG: sensors, application and future directions. *Artificial Intelligence: Theories and Applications. SETN*.

[12] Ali M., Mosa A. H., Al Machot F., Kyamakya K. EEG-based emotion recognition approach for e-healthcare applications.

[13] Zoubi O. A., Awad M., Kasabov N. K. (2018). Anytime multipurpose emotion recognition from EEG data using a Liquid State Machine based framework. *Artificial Intellingence in Medicine*.

[14] Nawaz R., Cheah K. H., Nisar H., Yap V. V. (2020). Comparison of different feature extraction methods for EEG-based emotion recognition. *Biocybernetics and Biomedical Engineering*.

[15] Craik A., He Y. T., Contreras-Vidal J. L. (2019). Deep learning for electroencephalogram (EEG) classification tasks: a review. *Journal of Neural Engineering*.

[16] Roy Y., Banville H., Albuquerque I., Gramfort A., Falk T. H., Faubert J. Deep learning-based electroencephalography analysis: a systematic review. *Journal of Neural Engineering*.

[17] Duan R.-N., Zhu J.-Y., Lu B.-L. Differential Entropy Feature for EEG-Based Emotion Classification.

[18] Zheng W.-L., Lu B.-L. (2015). Investigating critical frequency bands and channels for EEG-based emotion recognition with deep neural networks. *IEEE Transactions on Autonomous Mental Development (IEEE TAMD)*.

[19] Song T., Zheng W., Song P., Cui Z. (2018). EEG emotion recognition using dynamical graph convolutional neural networks. *IEEE Transactions on Affective Computing*.

[20] Lan Z., Sourina O., Wang L., Scherer R., Müller-Putz G. R. (2018). Domain adaptation techniques for EEG-based emotion recognition: a comparative study on two public datasets. *IEEE Transactions on Cognitive and Developmental Systems*.

[21] Li Y., Zheng W., Cui Z., Zong Y., Ge S. (2019). EEG emotion recognition based on graph regularized sparse linear regression. *Neural Processing Letters*.

[22] Wang Y., Qiu S., Li J. EEG-based emotion recognition with similarity learning network.

[23] Zhang T., Wang X., Xu X., Chen C. L. P., GCB-Net “ (2019). Graph convolutional broad network and its application in emotion recognition. *IEEE Transactions on Affective Computing*.

[24] Hwang S., Hong K., Son G., Byun H. (2019). Learning CNN features from DE features for EEG-based emotion recognition. *Pattern Analysis and Appliccations*.

[25] Zhang T., Cui Z., Xu C., Zheng W., Yang J. Variational pathway reasoning for EEG emotion recognition.

[26] Yang F., Zhao X., Jiang W., Gao P., Liu G. (2019). Multi-method fusion of cross-subject emotion recognition based on high-dimensional EEG features. *Frontiers in Computational Neuroscience*.

[27] Luo Y., Fu Q., Xie J. (2020). EEG-based emotion classification using spiking neural networks. *IEEE Access*.

[28] Eckart C., Young G. (1936). The approximation of one matrix by another of lower rank. *Psychometrika*.

[29] Maji P., Mullins R. (2018). On the reduction of computational complexity of deep convolutional neural networks. *Entropy*.

[30] Behncke J., Schirrmeister R. T., Burgard W., Ball T. The signature of robot action success in EEG signals of a human observer: decoding and visualization using deep convolutional neural networks.

[31] Chambon S., Galtier M. N., Arnal P. J., Wainrib G., Gramfort A. (2017). A deep learning architecture for temporal sleep stage classification using multivariate and multimodal time series. *IEEE Transactions on Neural Systems and Rehabilitation Engineering*.

[32] Kwak N. S., Müller K. R., Lee S. W. (2017). A convolutional neural network for steady state visual evoked potential classification under ambulatory environment. *PLoS One*.

[33] Manor R., Geva A. B. (2015). Convolutional neural network for multi-category rapid serial visual presentation BCI. *Frontiers in Computational Neuroscience*.

[34] Schirrmeister R. T., Springenberg J. T., Fiederera L. D. J. (2017). Deep learning with convolutional neural networks for EEG decoding and visualization. *Human Brain Mapping*.

[35] Zafar R., Dass S. C., Malik A. S. (2017). Electroencephalogram-based decoding cognitive states using convolutional neural network and likelihood ratio based score fusion. *PLOS ONE*.

[36] Cheah K. H., Nisar H., Yap V. V., Lee C.-Y. (2019). Convolutional neural networks for classification of music-listening EEG: comparing 1D convolutional kernels with 2D kernels and cerebral laterality of musical influence. *Neural Computing and Applications*.

[37] Ioffe S., Szegedy C. (2015). Batch normalization: accelerating deep network training by reducing internal covariate shift. https://arxiv.org/abs/1502.03167.

[38] Bjorck J., Gomes C., Selman B., Weinberger K. Q. (2018). Understanding batch normalization. https://arxiv.org/abs/1806.02375.

[39] Ansari-Asl K., Chanel G., Pun T. A channel selection method for EEG classificatoin in emotion assessment based on synchronization likelihood.

[40] Ozerdem M. S., Polat H. (2017). Emotion recognition based on EEG features in movie clips with channel selection. *Brain Informatics*.

[41] Zheng W.-L., Lu B.-L. (2015). Investigating critical frequency bands and channels for EEG-based emotion recognition with deep neural networks. *IEEE Transactions on Autonomous Mental Development*.

[42] Dolan R., Lane R., Chua P., Fletcher P. (2000). Dissociable temporal lobe activations during emotional episodic memory retrieval. *NeuroImage*.

[43] Dolcos F., LaBar K. S., Cabeza R. (2005). Remembering one year later: role of the amygdala and the medial temporal lobe memory system in retrieving emotional memories. *Preceedings of the National Academy of Sciences (PNAS)*.

[44] Iidaka T., Okada T., Murata T. (2002). Age-related differences in the medial temporal lobe responses to emotional faces as revealed by fMRI. *Hippocampus*.

[45] Corballis M. C. (2014). Left brain, right brain: facts and fantasies. *PLoS Biology*.

[46] Liu H., Stufflebeam S. M., Sepulcre J., Hedden T., Buckner R. L. (2009). Evidence from intrinsic activity that asymmetry of the human brain is controlled by multiple factors. *Preceedings of the National Academy of Sciences (PNAS)*.

[47] DeWitt I., Rauschecker J. P. (2013). Wernicke’s area revisited: parallel streams and word processing. *Brain and Language*.

